The article "Rethinking U-Net from an Attention Perspective with Transformers for Osteosarcoma MRI Image Segmentation" was published in 2022. Journal: Comput Intell Neurosci.

# Rethinking U-Net from an Attention Perspective with Transformers for Osteosarcoma MRI Image Segmentation

**DOI:** 10.1155/2022/7973404

**Published:** 2022-06-06

**Authors:** Tianxiang Ouyang, Shun Yang, Fangfang Gou, Zhehao Dai, Jia Wu

**Affiliations:** ^1^School of Computer Science and Engineering, Central South University, Changsha 410083, China; ^2^Department of Spine Surgery, The Second Xiangya Hospital, Central South University, Changsha 410011, China; ^3^Research Center for Artificial Intelligence, Monash University, Melbourne, Clayton, VIC 3800, Australia

## Abstract

Osteosarcoma is one of the most common primary malignancies of bone in the pediatric and adolescent populations. The morphology and size of osteosarcoma MRI images often show great variability and randomness with different patients. In developing countries, with large populations and lack of medical resources, it is difficult to effectively address the difficulties of early diagnosis of osteosarcoma with limited physician manpower alone. In addition, with the proposal of precision medicine, existing MRI image segmentation models for osteosarcoma face the challenges of insufficient segmentation accuracy and high resource consumption. Inspired by transformer's self-attention mechanism, this paper proposes a lightweight osteosarcoma image segmentation architecture, UATransNet, by adding a multilevel guided self-aware attention module (MGAM) to the encoder-decoder architecture of U-Net. We successively perform dataset classification optimization and remove MRI image irrelevant background. Then, UATransNet is designed with transformer self-attention component (TSAC) and global context aggregation component (GCAC) at the bottom of the encoder-decoder architecture to perform integration of local features and global dependencies and aggregation of contexts to learned features. In addition, we apply dense residual learning to the convolution module and combined with multiscale jump connections, to improve the feature extraction capability. In this paper, we experimentally evaluate more than 80,000 osteosarcoma MRI images and show that our UATransNet yields more accurate segmentation performance. The IOU and DSC values of osteosarcoma are 0.922 ± 0.03 and 0.921 ± 0.04, respectively, and provide intuitive and accurate efficient decision information support for physicians.

## 1. Introduction

Osteosarcoma is the most common malignant primary bone tumor, with the highest incidence among adolescents [1]. Among all children and adolescents, osteosarcoma accounts for the majority of diagnosed malignant bone tumors, approximately 55% [2]. Cancer deaths due to osteosarcoma account for up to 8.9% of all childhood and adolescent cancer deaths [3]. In addition, osteosarcoma is highly susceptible to pulmonary metastases if patients are not diagnosed and treated early. Studies have found that 46–66% of patients with osteosarcoma in developing countries already have metastatic disease at the time of presentation [4]. Osteosarcoma is characterized by high malignancy, aggressiveness, rapid disease progression, and high mortality and is considered a serious threat to human health worldwide.

For patients with osteosarcoma, if not diagnosed and treated early, there is a tendency to develop extensive metastases in other soft tissues [5]. In addition, no more than 20% of patients with advanced osteosarcoma survive longer than 5 years [6]. And, medical imaging is considered to be an important technique to help physicians assess the disease and optimize preventive and control measures [7]. To better plan patients' treatment plans, monitor changes in their condition, and perform prognosis, we often obtain valid information on osteosarcoma through medical image segmentation and quantitative assessment. Magnetic resonance imaging (MRI) has become a major tool for physicians to diagnose and evaluate osteosarcoma due to its absence of any ionizing radiation, safety and painlessness, low risk, and minimal harm to the body.

Most developing countries face a huge dilemma in the diagnosis and treatment of osteosarcoma. Take China as an example. China is a vast country with unbalanced medical development between regions, and the awareness of osteosarcoma is still unfamiliar in primary hospitals and even some provincial and municipal hospitals. And the occurrence, development, transformation, or deterioration of osteosarcoma are a dynamic process of change. With the different age, gender, physique, and even living conditions of patients, the morphology and size of osteosarcoma often show great variability and randomness. This places a high demand on the expertise of physicians. However, the poor and backward regions of China have poor medical equipment and shortage of professional physicians [8]. On the one hand, for atypical osteosarcoma conditions, physicians manually identify, segment, and diagnose them, which is prone to subjective assumptions and misdiagnosis. On the other hand, the total amount of redundant data in MRI images of osteosarcoma is huge and it is difficult to solve this problem effectively with limited physician manpower alone. These circumstances make early diagnosis and timely treatment of osteosarcoma in poor areas particularly difficult.

Modern medical imaging technology is developing rapidly, and computer-aided diagnosis (CAD) system is also constantly innovating. Sathiyamoorthi et al. [9] used adaptive histogram adjustment (AHA)-based algorithm for image enhancement to improve the image in terms of brightness and contrast. Gayathri et al. [10] have improved the accuracy of the model by using sparse self-encoder as a dimensionality reduction technique. CAD provides physicians with effective information to support disease treatment decisions, which to a certain extent alleviates the difficulties in early diagnosis of osteosarcoma caused by the shortage of specialized doctors in developing countries, and avoids misdiagnosis due to the time and effort spent by doctors in dealing with the complex diagnostic process and analyzing large amounts of case data. In recent years, machine learning has emerged and convolutional neural networks are widely used in image segmentation [11], and many full convolutional network (FCN)- [12] based methods have been proposed to accurately segment medical images. It can also be combined with squeeze-and-excitation (SE) block and multidataset training to improve the overall generalization ability of the model [13]. However, the low contrast between patient organs and blurred boundaries of osteosarcoma MRI images poses great difficulties for accurate detection and segmentation.

As the most popular encoder-decoder network in medical image segmentation [14], U-Net [15] segmented small targets better, had a scalable structure [16], and was widely used in osteosarcoma MRI image segmentation. However, as the performance requirement of medical image segmentation increases, U-Net shows the limitation of information decline due to the lack of ability to effectively construct remote feature dependencies and capture global contextual information. On the other hand, osteosarcoma MRI images are susceptible to noise and prone to overfitting resulting in edge feature loss.

Inspired by the self-attention mechanism of transformer [17], this paper proposes a lightweight osteosarcoma image segmentation architecture UATransNet by adding a multilevel guided self-aware attention module (MGAM) to the encoder-decoder architecture of U-Net. We successively perform dataset classification optimization and remove MRI image irrelevant backgrounds, reducing the waste of computational resources while optimizing the osteosarcoma segmentation performance. We designed two components: transformer self-attention component (TSAC) and global context aggregation component (GCAC). TSAC adaptively integrates local features with their global dependencies, and GCAC optimizes the effect of feature representation by aggregating contexts to learned features and better preserves detailed information such as osteosarcoma edge features. In this paper, we also apply dense residual learning [18] to the convolution module, combined with multiscale jump connection [19], to improve feature extraction. Meanwhile, the UATransNet method has few parameters, simple computation, and low hardware equipment requirements, which alleviates the difficulties of backward medical equipment in developing countries [20–25], achieves a balance of speed and accuracy, and greatly improves the diagnostic efficiency of physicians.

The detailed contributions of this study are as follows:

1. In this paper, we optimize the classification of dataset by mean-teacher model to alleviate the influence of noisy labels on model training; remove irrelevant backgrounds in osteosarcoma MRI images through dataset preprocessing to reduce the burden of input images on segmentation network; and then improve the accuracy and segmentation efficiency of osteosarcoma segmentation.
2. The incorporation of multilevel guided self-aware attention module (MGAM) into the encoder-decoder architecture of U-Net, which combines deep semantic information and spatial information through jump connections, provides the necessary fine-grained and high-resolution features for deconvolution, and facilitates the recovery of spatial information of osteosarcoma. In addition, the application of dense residual learning to the convolution module, combined with multiscale jump connections and aggregation of different semantic amplification sampling functions, facilitates the reduction of interference from osteosarcoma MRI image noise, and better preserves detailed information such as osteosarcoma edge features.
3. Two components, transformer self-attention component (TSAC) and global context aggregation component (GCAC), are designed in UATransNet to enhance the ability to construct remote feature dependencies and capture global contextual information. Among them, TSAC adaptively integrates local features with their global dependencies and GCAC optimizes the feature representation effect of osteosarcoma by aggregating contexts to learned features. Meanwhile, the UATransNet method has few parameters, simple computation, and low hardware equipment requirements, which alleviates the difficulties of backward medical equipment in developing countries and achieves a balance of speed and accuracy in osteosarcoma detection and segmentation, greatly improving the diagnostic efficiency of physicians.
4. Experimental analysis was performed using over 80,000 osteosarcoma MRI images acquired from Xiangya II Hospital of Central South University. Our proposed osteosarcoma image segmentation architecture exhibits better segmentation performance compared with some state-of-the-art baselines. Furthermore, it can enable the diagnostic accuracy of osteosarcoma images to approach the level of expert physicians, providing information support for decision-making in regions and countries lacking high-level physicians.

## 2. Related Work

Osteosarcoma is an aggressive malignant bone tumor that occurs mostly in the extremity bones of children and adolescents, with an extremely poor natural prognosis and a tendency to develop blood metastases at an early stage. Imaging is an important tool for the diagnosis and clinical evaluation of osteosarcoma. In recent years, computer-aided decision-making systems have become a popular research direction in the medical field to analyze the health status of patients mainly through healthcare data and diagnostic images.

Due to the cellular heterogeneity in the dataset, pathologists are often faced with high complexity processing and disagreement in classifying osteosarcoma tumors. Similarly, segmentation and classification of tissues in tumor images remain extremely challenging due to interclass similarity and intraclass variability, despite H&E staining. Chen and Zhao [26] proposed convolutional neural network (CNN) as a tool to improve the efficiency and classification of osteosarcoma into tumor categories (live tumor, necrosis) versus nontumor accuracy. Schlemper et al. [27] proposed a novel attention gate (AG) model for medical image analysis that can be easily integrated into standard CNN models, providing efficient object localization while incorporating manual annotations, which improves model sensitivity and prediction accuracy. To solve the problems of easy overfitting of models, weak image feature extraction, and low accuracy in automatic classification of surviving and necrotic tumor regions of osteosarcoma, Fu et al. [28] designed a deep model with a conjoined network (DS-Net) consisting of an auxiliary supervised network (ASN) and a classification network, which not only can effectively achieve histological classification of osteosarcoma but also can be applied to other medical image classification tasks that are affected by small datasets.

Various osteosarcoma detection methods are used for early detection of osteosarcoma, but evaluation of slides under the microscope to detect the extent of tumor necrosis and tumor outcome remains a major challenge in the medical field. Therefore, Badashah et al. [29] developed an effective detection method for early detection of osteosarcoma using the proposed fractional-Harris Hawks optimization-based generative adversarial network (F-HHO-based GAN). F-HHO was designed by integrating fractional calculus and HHO, while GAN extracted image features based on F-HHO algorithm and cell segmentation process, allowing better performance in terms of accuracy, sensitivity, and specificity. Currently, this evaluation is mainly done manually by pathologists observing slides under a microscope. However, the segmentation effect is limited due to the subjective nature of the manual operation. Ho et al. [30] proposed an effective labeling method for training CNNs, deep interactive learning (DiaL), where after the initial labeling step, the annotator simply corrects the mislabeled regions from the previous segmentation predictions to improve the CNN model until satisfactory predictions are obtained.

Diffusion-weighted imaging (DWI) can capture cellular changes in tumor tissue without contrast injection in the early stages of patient treatment, facilitating early diagnosis and prognosis of malignant disease [31]. Osteosarcoma has characteristics such as low signal-to-noise ratio and heterogeneous intensity, leading to great challenges in DWI tumor segmentation. To address the significant challenges of interpatient tumor variation and treatment option selection, Zhao et al. [32] combined radiological features extracted from diffusion-weighted magnetic resonance imaging (DWI-MRI) and traditional clinical features for osteosarcoma assessment to achieve better evaluation and could improve the prediction of overall survival for localized osteosarcoma. This approach may help to better select patients who are most likely to benefit from enhanced multimodal diagnosis and treatment.

In recent years, automatic segmentation based on deep learning has been widely used. Among them, U-Net is one of the most important semantic segmentation frameworks for convolutional neural networks (CNNs) and is widely used for lesion segmentation and classification in the field of medical image analysis. U-Net [33] is successfully used extensively in all major image modalities from CT scans to X-rays and even microscopy and plays an extremely important role, thus serving as the main tool in medical imaging segmentation tasks [34]. Shuai et al. [35] proposed a novel and more powerful architecture W-net++ based on two cascaded U-Net and dense skip connections. In this network, multiscale inputs are applied to the architecture to recover spatial details lost due to multiple encoding and secondary sampling of the encoder; adaptive depth supervision is introduced to guide multiscale learning of the network to accelerate convergence and improve network performance. It is also compared with the state-of-the-art method through a 5-fold cross-validation of a homemade osteosarcoma CT image dataset, which achieves automatic and more accurate segmentation of osteosarcoma lesions in computed tomography (CT) images.

In order to better extract edge features and texture features, etc. using the shallow edge output module, we extract semantic features using the deep output module, calculate the loss value between the predicted map and the actual tumor image by the side output module, and then backpropagate the loss information. Zhang et al. [36] proposed a multisupervised residual network for osteosarcoma image segmentation by adding three supervised side output modules to the residual network supervised residual network for osteosarcoma image segmentation. Then, the parameters of the residual network were modified by the gradient descent method, which in turn guided the multiscale feature learning of the network to obtain more accurate segmentation results.

Based on the above analysis, in order to better assist clinical diagnosis and treatment, the research on osteosarcoma image preprocessing, image segmentation, and image analysis by model construction has been developed significantly in recent years. However, the MRI images of osteosarcoma are susceptible to noise and have complex edge contours, making the segmentation effect poor. To optimize the segmentation effect of MRI images of osteosarcoma, we combine the depth-separable U-shaped network with transformer and propose a new perspective to improve the performance of semantic segmentation, which achieves more effective feature fusion by multilevel guided attention, i.e., collaborating with transformer's self-attention and global spatial attention, and multiscale exploration of connected contextual semantic information to ensure the semantic embedding consistency.

## 3. Methods

### 3.1. Overview of UATransNet

With the development of intelligent medicine, image processing plays an indispensable role in the diagnosis, treatment, and prognosis of diseases. Osteosarcoma MRI images have complex features and contain a lot of redundant data, which makes manual screening and detection by physicians alone time-consuming and laborious. U-Net is widely used for MRI image segmentation of osteosarcoma because of its better segmentation of small targets and scalable structure. However, as the performance requirement of medical image segmentation increases, U-Net shows the limitation of information decline due to the lack of ability to effectively construct remote feature dependencies and capture global contextual information. On the other hand, osteosarcoma MRI images are susceptible to noise and prone to overfitting resulting in loss of edge features. Based on this, we propose a lightweight UATransNet osteosarcoma image segmentation model by combining the encoder-decoder architecture of U-Net with transformer. We successively perform dataset classification optimization and remove irrelevant backgrounds from MRI images by averaging teacher models and normalizing preprocessing. In order to break the limitation of information degradation exhibited by U-Net due to the lack of ability to effectively construct remote feature dependencies and capture global contextual information, we designed two components: transformer self-attentive component (TSAC) and global contextual aggregation component (GCAC). TSAC adaptively integrates local features with their global dependencies to better preserve osteosarcoma edge features and other detailed information, and GCAC optimizes the osteosarcoma feature representation by aggregating context to the learned features.

In addition, this paper applies dense residual learning to the convolution module, combined with multiscale jump junction, to improve the feature extraction capability. Using over 80,000 osteosarcoma MRI images acquired at Xiangya II Hospital of Central South University for experimental analysis, our proposed osteosarcoma image segmentation architecture exhibits better segmentation performance compared to some state-of-the-art baselines. In addition, the diagnostic accuracy of osteosarcoma images is close to that of expert physicians, providing intuitive and accurate information support for decision-making in regions and countries that lack high-level physicians.

In this section, the proposed UATransNet model is introduced in terms of dataset optimization, normalized preprocessing, multilevel guided attention mechanism, and multiscale jump connection. The overall design of the proposed UATransNet osteosarcoma image segmentation model in this paper is shown in Figure 1.

### 3.2. Dataset Optimization

We selected over 80,000 osteosarcoma MRI images as the dataset for our experiments, but among them, some of the images had too small or blurred osteosarcoma regions, which led to significant degradation of the experimental model performance. To improve the accuracy of the test, we combined the mean-teacher network [37], ResNet [38], and residual learning to optimize the classification of the initial dataset before the model experiment.

To cope with the possible gradient disappearance problem as the number of network layers increases, we use residual connections and three 3 × 3 convolutional blocks to capture the high-dimensional feature information of the image and use group normalization instead of batch normalization in the Res-Block to cope with the possible performance degradation caused by small batches, as shown in Figure 2, where the Res-Block consists of convolutional layers, GN, and residual connections. Then, 6-layer Res-Block is then used to combine the maximum pooling layer to simultaneously reduce the effect of feature maps. Finally, the dataset is classified by a fully connected layer and the whole architecture acts as a teacher model as well as a student model.

First, we randomly divide the original dataset into two parts, *D*_1_ and *D*_2_. Among them, the *D*_1_ dataset contains *Label*_1_ and the *D*_2_ dataset does not contain the label. The overall design of the mean-teacher semisupervised algorithm is shown in Figure 3.

Mean-teacher semisupervised algorithm: first, the *D*_1_ and *D*_2_ datasets are input to the student model, and the predicted likelihood of *P*_*stu*  *de*  *nt*1_ and *P*_*stu*  *de*  *nt*2_ is output; the *D*_2_ dataset is input to the teacher model, and the predicted likelihood *P*_*teacher*2_ is output. Second, the loss value *V*_1_ is calculated based on the loss function *Loss*_1_ and *P*_*stu*  *de*  *nt*1_ and *P*_*teacher*1_ can calculate the loss value *V*_1_, which is calculated as follows [39]:

(1) $$\begin{array}{c} Loss_{1}=-\frac{1}{n}\overset{n}{\underset{t=0}{\sum }}l_{t}\cdot \;\log\left(p_{t}\right)+\left(1-l_{t}\right)\cdot \;\log\left(1-p_{t}\right),l_{t}\in Label_{1},p_{t}\in P_{stu\;de\;nt1}. \end{array}$$

Similarly, the loss value *V*_2_ is calculated based on the loss function *Loss*_2_ and *P*_*stu*  *de*  *nt*2_ and *P*_*teacher*2_. The network parameters of the teacher model of UATransNet  *θ*_*t*_′ are obtained by updating the network parameters of the student model  *θ*_*t*_ by moving average.

(2) $$\begin{array}{c} \theta_{t}^{\prime }=\alpha \theta_{t-1}^{'}+\left(1-\alpha \right)\theta_{t}. \end{array}$$

The network parameters *θ*_*t*_ of student model are obtained by updating the parameters through loss gradient descent. Among them, the loss function contains two parts: the first part is the supervised loss function, as shown in equation (1). *Loss*_1_ is the cross-entropy loss function, which mainly ensures the labeled training data fit; the second part is the unsupervised loss function, which uses the Kullback–Leibler (KL) scattering relative entropy loss function [40]; the KL formula is shown as follows. Its main purpose is to ensure that the prediction results of the teacher network are as similar as possible to the prediction labels of the student network.

(3) $$\begin{array}{c} Loss=Loss_{1}+Loss_{2},\\ KL\left(Q\mathrm{||}P\right)=\sum p\left(x\right)\cdot \;\log\frac{p\left(x\right)}{q\left(x\right)}. \end{array}$$

However, there is a problem of asymmetry in the KL function. In order to make the prediction distribution of the teacher model and the student model consistent, we adopted the Jensen–Shannon (JS) algorithm [41] to compensate for the asymmetry problem, so *Loss*_2_ is calculated as follows:

(4) $$\begin{array}{c} Loss_{2}=\frac{1}{2}KL\left(P_{stu\;de\;nt2}\left\|P_{teacher2}\right.\right)+\frac{1}{2}KL\left(P_{teacher2}\|\left\|P_{teacher2}\right.\right). \end{array}$$

Finally, we divided the osteosarcoma MRI image dataset into effective part and difficult part with the proportion of 39.4% and 60.6%, respectively, and input them into the UATransNet network model sequentially to achieve better training effect.

### 3.3. Pretreatment

To remove irrelevant backgrounds from the osteosarcoma MRI images and reduce the burden of the input images on the network, we segmented the input osteosarcoma MRI images into osteosarcoma-suspected regions and the processing steps are shown in Figure 4. The threshold value is adaptively adjusted according to the size of the osteosarcoma to prevent undersegmentation or oversegmentation [42].

#### 3.3.1. Region-of-Interest Detection

First, a multiscale deep belief network (m-DBN) and Gaussian mixture classifier (GMC) [43] were used to extract suspicious regions, and a rectangular boundary of a larger suspected region of osteosarcoma was framed as an input.

#### 3.3.2. Image Preprocessing

In the image matrix, the minimum weight of histogram is 5%. The upper bound and the next bound of the adjusted weight are less than 5%. The image is then median filtered to remove noise using a window of a certain size, which is 5% of the maximum value of the length height of the region of interest. However, since the use of median filtering [44] leads to the generation of false contours, to protect the image edges, mean filtering is used to reduce the effect of false contours. Finally, a Laplace filter with the same window size is used to enhance the edges of the region of interest.

#### 3.3.3. Osteosarcoma Size Estimation

The Otsu method [45] was used to generate two regions based on the intensity histogram of the image: the larger region and the smaller region. In this way, the size of the osteosarcoma can be roughly estimated as larger than the smaller region and smaller than the larger region. Also, the segmentation point of the intensity histogram generated by the Otsu method will be used as the threshold for the fourth step of the seed region growth algorithm.

#### 3.3.4. Suspected Area Segmentation

Based on a priori knowledge, in osteosarcoma MRI images, the tumor region is generally brighter than the surrounding healthy tissue. Therefore, the brighter multiple pixel points in the center of the region of interest are selected as the initial seed points. The following two principles are followed when selecting the pixel points adjacent to the seed points to be added to the seed points:

(5) $$\begin{array}{c} \left|\mu -I_{x^{\prime },y^{\prime }}\right|<\theta ,\\ I_{x^{\prime },y^{\prime }}>\theta , \end{array}$$

where *μ* is the average intensity of the image pixels in the segmented region, *I*_*x*′,*y*′_ is the intensity of the candidate pixel points located at (*x*′, *y*′), and *θ* is the determined threshold. Then, the threshold value obtained in the third step of osteosarcoma size estimation is used as the initial threshold value, and when no remaining pixels satisfy the seed expansion conditions specified by the above two equations, the size of the segmented region obtained in the current evolutionary stage is checked in relation to the predicted osteosarcoma size; if the currently obtained region size is smaller than the estimated value, the threshold value is lowered to continue expanding the region; if the currently obtained region is larger than the estimated value, the segmentation is stopped.

The threshold is adjusted adaptively according to the size of the osteosarcoma, and the input osteosarcoma MRI image is segmented into the suspected region of the osteosarcoma. The grayscale characteristics of the image can be directly used, the calculation is simple, and the calculation efficiency is high, but for a few grayscale differences that are not obvious, images with a large disparity in the size and proportion of the target and the background, you need to combine manual experience selection to have a better effect. Therefore, this paper mainly focuses on most of the MRI images of osteosarcoma with obvious gray difference.

### 3.4. Multilevel Guided Attention Mechanism (MGAM)

The U-Net network model for segmenting osteosarcoma MRI images is able to fuse deep semantic information (such as the color and shape of the osteosarcoma) with the information contained in high-precision features but is unable to model the contextual relationships of features that are far away, resulting in insufficient accuracy for osteosarcoma segmentation. Like the opposite, the transformer network model employs a self-attentive mechanism, which facilitates the extraction of global information but lacks information at local details. Based on this, we propose a lightweight UATransNet osteosarcoma image segmentation model with a multilevel guided self-aware attention module (MGAM) between the bottom encoder and decoder of the U-shaped architecture, which helps to capture a broader and richer contextual representation and better fuses the features of semantic inconsistency between transformer and U-Net network models. It is beneficial to reduce the interference of osteosarcoma MRI image noise, so that detailed information such as osteosarcoma edge features is better preserved and excellent segmentation results can be obtained. In addition, represented by MGAM, UATransNet has a small number of parameters and simple computation, which reduces the consumption of resources and achieves a balance of accuracy and efficiency of osteosarcoma MRI image segmentation.

The core component of the UATransNet proposed in this paper: the multilevel guided self-aware attention module (MGAM) consists of the transformer self-attention component (TSAC) and the global context aggregation component (GCAC).

#### 3.4.1. Transformer Self-Attention Component (TSAC)

Referring to transformer's multihead self-attention mechanism, UATransNet focuses on semantic information from the global contextual representation subspace and first adds the learned position encoding of the osteosarcoma MRI image to the input of the encoder features and shares it among all attention layers for a given query/key value sequence, enabling the capture of contextual information about absolute and relative positions [46], which is then computed separately in multiple single attention heads and combined by another embedding.

The concrete implementation of the TSAC is shown in Figure 1. The encoder feature Feature Map ∈*R*^*c*×*h*×*w*^ as input is first reconstructed as a query matrix *Q* ∈*R*^*c*×(*h* × *w*)^ and key matrices *K* ∈*R*^*c*×*h*×*w*^ and *V* ∈*R*^*c*×*h*×*w*^ [47], and the *Q*, *K*, and *V* matrices contain the texture features of the osteosarcoma MRI image.

(6) $$\begin{array}{c} Q=Feature\cdot W_{q},\\ K=Feature\cdot W_{k},\\ V=Feature\cdot W_{v}, \end{array}$$

where *W*_*q*_, *W*_*k*_, and *W*_*v*_ are embedding matrices for different linear projections. Then, a scaled dot product operation with softmax normalization between the transposed versions of the query and key matrices is used to generate a matrix of contextual attention maps CAM ∈*R*^*c*×*c*^ and captures the necessary fine-grained and high-resolution features in the osteosarcoma MRI images. The matrix exhibits similarity to the global elements of the key matrix compared to the given elements from the query matrix. To further implement the aggregation of values weighted by attention weights, we multiplied the contextual attention map CAM by *V* and recovered the detailed information in the osteosarcoma MRI images. Finally, in the TSAC, we can represent the multiheaded attention as follows:

(7) $$\begin{array}{c} \text{TSAC}\left(Q,K,V\right)=\text{soft}\max\left(\frac{Q\cdot K^{T}}{\sqrt{d_{k}}}\right)V. \end{array}$$

It should be noted that $\sqrt{d_{k}}$ is the dimension of the query/key sequence in equation (6). Finally, the feature map of the osteosarcoma MRI image obtained by our dot product operation optimization is also the final output of the transformer self-attention component (TSAC) part.

#### 3.4.2. Global Context Aggregation Component (GCAC)

UATransNet encodes broader contextual location information into local features via GCAC and selectively aggregates global context into the learned features. The specific implementation is shown in Figure 1. This not only optimizes the feature representation and helps to reduce the interference of osteosarcoma MRI image noise but also improves the intraclass compactness and facilitates the recovery of spatial information of osteosarcoma.

UATransNet first generates the feature maps *Feature*_*p*_^*c*_0_^ ∈ *R*^*c*_0_×*h*×*w*^ and *Feature*_*p*_^*c*_1_^ ∈ *R*^*c*_1_×*h*×*w*^, where *c*_1_=*c*_0_/8, respectively, using two convolution operations via the encoder feature *Feature*_*enco*  *de*  *r*_. Then, *Feature*_*p*_^*c*_0_^ is reshaped into *U*_*p*_^*c*_0_^ ∈ *R*^*c*_0_×(*h* × *w*)^ and *Feature*_*p*_^*c*_1_^ is reshaped into *V*_*p*_^*c*_1_^ ∈ *R*^*c*_1_×(*h* × *w*)^ and *W*_*p*_^*c*_1_^ ∈ *R*^*c*_1_×(*h* × *w*)^. Next, the matrix multiplication operation with softmax normalization is executed on the reshaped V and W to obtain the position attention map *L* ∈ *R*^(*h* × *w*)×(*h* × *w*)^:

(8) $$\begin{array}{c} L_{i,j}=\frac{\exp\left(V_{i}\cdot W_{j}\right)}{\sum_{i=1}^{n}\exp\left(V_{i}\cdot W_{j}\right)}, \end{array}$$

where *L*_*i*,*j*_ measures the effect of the ith location on the jth location and *n* = *h* × *w*, where *n* is the number of pixels in the osteosarcoma MRI image. Then, *L* is reshaped and multiplied with *W*, and the feature results for each location can be expressed as

(9) $$\begin{array}{c} GCAC{\left(U,V,W\right)}_{j}=\overset{n}{\underset{i=1}{\sum }}\left(L_{i,j},W_{j}\right). \end{array}$$

Finally, the feature results are reshaped to obtain the final output of the global context aggregation component (GCAC).

In order to fully utilize the obtained contextual information and spatial relationships, the multilevel guided self-aware attention function module takes a dynamic planning approach to optimally combine the original features and attention feature embeddings of osteosarcoma through attention embedding fusion, which is the important reason why UATransNet can acquire spatial information of osteosarcoma and accurately segment the MRI images of osteosarcoma.

(10) $$\begin{array}{c} Feature_{MGAM}=\propto_{1}Feature_{TSAC}+\propto_{2}Feature_{GCAC}+Feature_{enco\;de\;r}, \end{array}$$

where ∝_1_ and ∝_2_ are scale parameters initialized to 0. In this way, we can further optimize the feature representation of osteosarcoma MRI images with semantic consistency to obtain more accurate segmentation of osteosarcoma MRI images and provide intuitive, accurate, and efficient decision information support for physicians.

### 3.5. Multiscale Skip Connections

In this paper, feature maps from all scales are directly connected to form a unified tensor through cascade connection, and then, the features of the target are extracted, as shown in Figure 5. Specifically, the feature maps from different semantic scales of the osteosarcoma MRI images are first upsampled to a common resolution by bilinear interpolation; then, they are all directly connected to form a unified feature representation, which is expressed by the following equation:

(11) $$\begin{array}{c} F=f\left(v\left(F_{1}\right)v\left(F_{2}\right)\cdots v\left(F_{n}\right)\right), \end{array}$$

where *υ* (·), ⊕, and *f* (·) are the upsampling, concatenation, and mixed convolution operations, respectively.

The higher-level network has a larger perceptual field with strong semantic information representation capability; however, this structure results in low resolution of feature and lacks spatial geometric feature details; the lower-level network has a smaller perceptual field with strong geometric detailed information representation capability and weak semantic information representation capability though high resolution. In order to fuse multiscale features to be equally effective in encoding global and local contexts, UATransNet guides the upsampling process in the decoder subnetwork through a new multiscale jump connection scheme, i.e., residual connection and dense connection, and the network structure is shown in Figure 6. UATransNet is the decoder subnetwork, through a series of upsampling, connection, and convolution transformation operations to aggregate residual or dense features at different semantic scales to segment tumor regions of different sizes at multiple scales, thus improving the semantic segmentation accuracy of osteosarcoma.

#### 3.5.1. Residual Connection

As an input module, the model improves the structure of MRI images of osteosarcoma and solves the problem of unbalanced classification of MRI images of osteosarcoma (10).

(12) $$\begin{array}{c} F=f_{n}\left(F_{n-1}\right)v_{n}\left(F_{n-1}\right). \end{array}$$

#### 3.5.2. Dense Connection

To cope with the medical dilemma of outdated hardware equipment in developing countries, UATransNet employs a dense connection module in the encoder-decoder architecture. Dense concatenation takes the upsampled feature set of the previous encoder block as the input to the current block and the output feature map as the input to all subsequent blocks, as expressed in the upcoming equation. One advantage of dense connectivity is that it has fewer parameters than traditional convolutional networks because it does not need to relearn redundant feature maps, reducing the requirement for hardware equipment and alleviating the difficulties of poor medical equipment in poor areas.

(13) $$\begin{array}{c} F_{n}=f_{n}\left(\left[v_{n}\left(F_{0}\right)v_{n}\left(F_{1}\right)\cdots v_{n}\left(F_{n-1}\right)\right]\right). \end{array}$$

UATransNet aggregates multiple decoder features at different semantic scales by bilinear interpolation, which better preserves detailed information such as osteosarcoma edge features. In addition, the dense concatenation mechanism generates the most discriminative feature representation in contrast to using one-time cascade concatenation. In these ways, the UATransNet osteosarcoma image segmentation model can not only mitigate the loss of details due to excessive upsampling but also alleviate the problems of gradient disappearance and overfitting.

UATransNet successively performs dataset classification optimization and removes MRI image irrelevant background by averaging the teacher model and normalized preprocessing, which reduces the waste of computational resources, reduces the requirement for hardware devices, and greatly improves the efficiency of osteosarcoma segmentation. Then, UATransNet integrates local features and global dependencies in TSAC and GCAC at the bottom of the encoder-decoder architecture, which effectively reduces the interference of osteosarcoma MRI image noise. In addition, UATransNet applies dense residual learning to the convolution module and combines multiscale jump connections to better retain detailed information such as osteosarcoma edge features, which can provide doctors with fast and accurate decision suggestions, effectively simplify the diagnosis process, save time, and reduce the burden of tedious medical work for doctors.

## 4. Experiments

### 4.1. Dataset

The dataset used in the experiment is over 80,000 osteosarcoma MRI images and related indexes of 286 osteosarcoma patients in Xiangya II Hospital of Central South University in recent years provided by the Ministry of Education Mobile Health Information-China Mobile Joint Laboratory and Xiangya II Hospital of Central South University [1]. In order to better evaluate the semantic segmentation effect of the model on osteosarcoma images in the experiment, we performed data enhancement by rotating the images by 90°, 180°, and 270° and then put them into the same network segmentation to enhance the generalization ability of the model. There are 286 cases in this experimental dataset, and we roughly divide them into training and testing sets by 7 : 3, respectively. Considering the variability of osteosarcoma morphology and segmentation difficulty of patients in different age groups, we took age as the main information item and selected 75.52% of the data, i.e., 216 cases, as the training set, and 24.48%, i.e., 70 cases, as the test set randomly, based on the principle that the approximate proportion of training and test sets were drawn from the same age group. Patient-related information is shown in Table 1.

### 4.2. Baselines

In our experiments, we applied two different approaches to implement UATransNet, UATransNet Residual, and UATransNet Dense osteosarcoma segmentation models based on residual connections and dense connections, respectively. In addition, we also used a wide range of algorithms such as U-Net, PSPNet [48], MSFCN [49], MSRN [50], FCN, and FPN [51] as baselines and our proposed UATransNet Residual and UATransNet Dense for comparative experimental analysis. A brief description of these baseline models is given as follows:

1. U-Net: the U-structure U-Net combines deep semantic information and spatial information through skip connections of the encoder and decoder, providing necessary high-resolution features for deconvolution, which is beneficial to recover valuable spatial information
2. The core of pyramid scene parsing network (PSPNet): PSPNet aggregates contextual information from different regions to obtain global information through the pyramid pooling module
3. MSFCN: based on a fully convolutional network, multiscale feature learning is performed with three supervised output layers, and both local and global features are captured
4. Multiscale residual network (MSRN): convolutional kernels of different sizes are introduced for adaptive detection of image features at different scales
5. Fully convolutional network: FCN classifies images at the pixel level and uses a jump structure to achieve fine segmentation
6. Feature pyramid network (FPN): both high-resolution features in the lower layers and high semantic information features in the higher layers are fused and predicted separately for each fused feature layer

### 4.3. Implementation Details and Evaluation Metrics

UATransNet was implemented using PyTorch, Cuda 11.3, and all experiments were run on 1 RTX A4000 GPU with 32 G of memory. Before training the UATransNet model, we extended the dataset by scaling up (scaling down) images, rotating images, and flipping images to enhance the robustness of the model. During training, our proposed UATransNet framework was trained for 100 epochs with an initial learning rate set to 0.001, which changed to 0.0001 when training reached 50 epochs and was dynamically adjusted using CosineAnnealingLR. Through experiments, it can be seen that each epoch in the training process takes about 1–5 minutes. Finally, 100 epochs of verification are performed using the checkpoints that store the trained models, and the changes in the evaluation metrics for each epoch are recorded. The verification time of each epoch is about 6–10 s. In the process of parameter adjustment, we mainly set different parameter combinations such as ∝_1_=1, ∝_2_=0, ∝_1_=0.75, ∝_2_=0.25, ∝_1_=0, ∝_2_=1, ∝_1_=0.5, ∝_2_=0.5, ∝_1_=0.25,  and ∝_2_=0.75 by setting different ∝_1_ and ∝_2_ values and observe PRE, IOU, DSC, and other changes in the evaluation indicators to find the parameter combination with the best performance of the model.

To measure the similarity between the predicted mask and ground truth, we used accuracy (ACC), precision (PRE), recall (REC), dice similarity coefficient (DSC), intersection over union (IOU), and F1-score (F1) as measures, which were calculated in pixels and used to quantitatively evaluate the performance of the UATransNet model for osteosarcoma image segmentation. The specific definitions of each indicator are as follows:

(14) $$\begin{array}{c} \text{ACC}=\frac{\text{TP}+\text{TN}}{\text{TP}+\text{TN}+\text{FP}+\text{FN}}\text{,}\\ \text{PRE}=\frac{\text{TP}}{\text{TP}+\text{FP}}\text{,}\\ \text{REC}=\frac{\text{TP}}{\text{TP}+\text{FN}}\text{,}\\ \text{IOU}=\frac{\text{TP}}{\text{TP}+\text{FP}+\text{FN}}\text{,}\\ \text{DSC}=\frac{2*\left|I_{1}\cap I_{2}\right|}{\left|I_{1}\right|+\left|I_{2}\right|},\\ \text{F}1=\frac{2\cdot \text{PRE}\cdot \text{REC}}{\text{PRE}+\text{REC}}. \end{array}$$

### 4.4. Evaluation of Segmentation Effect

In the UATransNet osteosarcoma image segmentation model, we first perform classification optimization of the dataset, as shown in Figure 5, and we classify the dataset with small osteosarcoma area and blurred boundaries between osteosarcoma tissue and normal tissue, which require a lot of computational power in the training process, as the difficult part, and the dataset with clear outline of osteosarcoma image as the effective part. We input the classification-optimized and unprocessed datasets into the UATransNet osteosarcoma image segmentation model to obtain the respective model segmentation results, as shown in Figure 7. It is obvious that the completeness and accuracy of the prediction results from the classification-optimized dataset are significantly higher than those from the unprocessed dataset directly into the segmentation model and are highly similar to the true labels. This shows that the performance of the model has been significantly improved after the optimization of the dataset. As shown in Tables 2 and 3, comparing the confusion matrix values of a certain validation process of the classification model before and after dataset preprocessing, it can be seen that by optimizing the composition of the dataset and improving the effectiveness of image input, the ratios of TP and TN have been greatly increased, an increase of 17.7% and 37.5%, respectively.

Figure 8 shows the results of segmentation of MRI images of osteosarcoma by each model. As shown in the figure, it can be found that our UATransNet can detect and retain detailed information such as edge contours of osteosarcoma images more effectively than other baselines; thus, the segmentation accuracy of osteosarcoma MRI images is higher and best meets the segmentation criteria, and the segmentation output approximates the underlying facts.

In order to evaluate the performance of different osteosarcoma segmentation models more clearly and accurately, we performed a quantitative representation of the segmentation effect. We tested by training with 100 epochs, using accuracy (ACC), precision (PRE), recall (REC), dice similarity coefficient (DSC), intersection over union (IOU), and F1-score (F1) as measures for comparative analysis. The comparative results of the evaluation metrics are shown in Table 4.

As shown in Table 4, it can be seen that each baseline model performs with its own advantages and disadvantages. Among them, U-Net has a small number of parameters and low spatial complexity, which is more conducive to the training process, but the recall standard deviations are large and easy to miss; PSPNet has a small FLOPS, which can save a lot of computational cost in MRI image segmentation, but the segmentation performance of this model is less satisfactory; MSFCN and MSRN have good performance in each segmentation index, and their FLOPS values are as high as 1524.34 G and 1461.23 G, respectively, which occupy too much space; similarly, the parameters of FCN-16s and FCN-8s are too large, which is not conducive to model training. Finally, the FPNs with the best overall performance in the baseline model have relatively large standard deviations for each segmentation metric, and the confidence level is not sufficient.

However, our proposed UATransNet Residual and UATransNet Dense showed good performance in the osteosarcoma image segmentation task, and both models outperformed other baseline models in accuracy (ACC), precision (PRE), recall (REC), intersection over union (IOU), dice similarity coefficient (DSC), and F1-score(F1). UATransNet Residual and UATransNet Dense not only greatly optimize the segmentation accuracy, but also their FLOPs were only 161.01G and 163.20G, respectively, as shown in Figure 9, which achieved the accuracy-velocity-space occupation balance while greatly improving the segmentation accuracy, providing a new solution for accurate segmentation of osteosarcoma in developing countries. In addition, because UATransNet Dense uses dense connections, which may lead to a large amount of redundant information, and the F1-score of UATransNet Residual is about 0.53% higher than that of UATransNet Dense, showing a more sensitive diagnostic sensitivity and smaller and more stable standard deviations.

As shown in Figure 10, the results showed that our proposed UATransNet osteosarcoma segmentation model performed well in terms of accuracy, with UATransNet Residual and UATransNet Dense achieving 96.2% and 96.0% accuracy for osteosarcoma segmentation, respectively; especially, UATransNet Residual was better than the other baseline models in FCN-8s, which had the highest accuracy, and was still 2.23% higher. In addition, the precision of the UATransNet osteosarcoma segmentation architecture was higher than the other four comparison baselines in almost all of the 100 epochs and maintained at a high level. On the other hand, the parametric numbers of UATransNet Residual and UATransNet Dense are 17.9M and 18.3M, respectively, which are maintained at a lower level and are more favorable for the training process, as shown in Figure 11. In addition, for medical image semantic segmentation, it is most important to achieve accurate segmentation and prediction, which will directly affect the clinician's diagnosis of the condition and the decision of the treatment plan. The performance of UATransNet Residual and UATransNet Dense is excellent, with DSC values of 0.921 and 0.916, respectively, far exceeding other baselines, providing intuitive and accurate information to support physicians in developing countries.

For medical disease detection, if the recall rate is low, a bad situation such as a missed diagnosis can easily occur. Therefore, we pay particular attention to the analysis of the recall rate when we evaluate the performance of the osteosarcoma image segmentation model. In this experiment, we compared the recall rate of the UATransNet model with other baseline models, as shown in Figure 12. As can be seen from the chart, the recall rate of U-Net, FPN, and MSFCN models fluctuated greatly in the early stage of training. And the data of MSRN model fluctuate during the training process. However, the UATransNet model has maintained a higher recall rate than the other baseline models throughout the experiment.

In addition, we carefully analyzed how the accuracy of UATransNet and the individual baseline models changed with the progression of 100 epochs, as shown in Figure 13. In the later stage of training, the accuracy of each model stabilized between a certain range of values. Among them, UATransNet has the highest accuracy rate of 99.1%. And, the accuracy of UATransNet osteosarcoma segmentation architecture shows excellent stability during the training process of 100 epochs, which is basically higher than 95%, so it can be seen that the segmentation prediction results obtained by UATransNet are closer to the real results compared with other baseline models. The prediction results obtained by UATransNet are closer to the real results than other baseline models. Finally, the ranking of each baseline model for osteosarcoma image segmentation is as follows: UATransNet > U-Net > FPN > FCN-8s ≈ FCN-16s > MSRN > MSFCN.

The F1-score is a statistical measure of the accuracy of a binary classification model. It takes into account both the accuracy and recall of the classification model. As can be seen from Figure 14, after 100 epochs of training, the F1-score of UATransNet finally stabilized at around 95%, showing better robustness among the various osteosarcoma segmentation models. As the average value of the reconciliation of precision and recall, the F1-score taken as high as 95.5% fully illustrates the good segmentation performance of UATransNet on osteosarcoma MRI images.

## 5. Discussion

Osteosarcoma MRI image segmentation helps physicians in clinical diagnosis by providing precise contours of osteosarcoma and assisting them in the clinical process. We designed a novel network, UATransNet, based on a modified U-Net, by introducing a self-attentive mechanism, incorporating a self-aware attention module, and combining it with a mean-teacher model, which produced good segmentation performance with IOU and DSC of 0.922 ± 0.03 and 0.921 ± 0.04, respectively. To further explore the effectiveness of MRI image segmentation in supporting the neuro-radiosurgery treatment planning stage, Rundo et al. [52] and Militello et al. [53] used a semiautomatic segmentation method based on an unsupervised fuzzy C-mean clustering algorithm for brain tumor necrosis identification study. On the one hand, their method achieves lesion volume measurement; on the other hand, the method evaluates based on spatial overlap and distance-based metrics with strong robustness while still having good segmentation performance and a DSC value of 95.93 ± 4.23. However, each patient still generates a large number of MRI images in a single diagnosis, resulting in a large consumption of computational resources. In contrast, UATransNet has a small number of parameters and simple computation, which achieves a balance of image segmentation accuracy and efficiency and provides a new solution idea for other organs to perform necrosis detection.

## 6. Conclusions

This paper proposes a novel lightweight osteosarcoma image segmentation model, UATransNet, based on over 80,000 osteosarcoma image datasets collected from Xiangya II Hospital of Central South University for extensive experiments. UATransNet significantly improves the accuracy of osteosarcoma segmentation based on the original computational power through dataset classification optimization and preprocessing, and achieves the trade-off between accuracy and speed; utilizes TSAC and GCAC components are used to optimize the feature representation effect of osteosarcoma; applying dense residual learning to the convolution module, combined with multiscale jump junction, better preserves the edge features of osteosarcoma, provides effective decision information support for clinicians, and provides a new option for early diagnosis and treatment of osteosarcoma in developing countries.

However, this paper is not clear enough for edge segmentation of osteosarcoma MRI images with little grayscale difference. With the development of medical image segmentation technology, in future research work, we will comprehensively utilize and optimize the edge features and texture features of osteosarcoma MRI images to further optimize the segmentation effect of osteosarcoma MRI images.

## Figures and Tables

**Figure 1:** Illustration of the UATransNet medical image segmentation framework for osteosarcoma MRI. Among them, UATransNet successively performs dataset classification optimization and removes MRI image irrelevant background by averaging teacher models and normalized preprocessing. Then, UATransNet is designed with transformer self-attention component (TSAC) and global context aggregation component (GCAC) at the bottom of the encoder-decoder architecture to perform integration of local features and global dependencies and aggregation of contexts to learned features.

**Figure 2:** The left side of the figure is the architectural design of the student model/teacher model, and the right side is the overall architecture of Res-Block consisting of convolutional layers, GN, and residual connections.

**Figure 3:** Optimization process of the osteosarcoma MRI image dataset based on mean-teacher semisupervised algorithm.

**Figure 4:** The input osteosarcoma MRI image is segmented into the suspected area of osteosarcoma to remove the irrelevant background in the osteosarcoma and reduce the network burden.

**Figure 5:** Cascade connections connect feature maps from all scales to form a unified tensor through operations such as upsampling, concatenation, and hybrid convolution.

**Figure 6:** Residual connections connect the input and output features of each decoder block as input to subsequent blocks. Dense connections work by taking the upsampled features of previous decoder blocks as input and feeding their own feature maps into all subsequent blocks together.

**Figure 7:** The prediction results after dataset optimization and input into the segmentation model are significantly better than the direct input into the segmentation model and are highly close to the labeled values.

**Figure 8:** Examples of the effect of osteosarcoma segmentation with UATransNet and different advanced baseline models on the test dataset and the DSC values of the corresponding predicted images.

**Figure 9:** FLOPs for UATransNet and different advanced baseline models.

**Figure 10:** Comparison of the UATransNet osteosarcoma segmentation model with other baselines in terms of precision performance.

**Figure 11:** Comparison of parameters of UATransNet and different advanced baseline models and DSC values of predicted images on the test dataset.

**Figure 12:** Comparison of the UATransNet osteosarcoma segmentation model with other baselines in terms of recall performance.

**Figure 13:** Comparison of the UATransNet osteosarcoma segmentation model with other baselines in terms of accuracy performance.

**Figure 14:** Comparison of the UATransNet osteosarcoma segmentation model with other baselines in terms of F1-score performance.

**Table 1:** The baseline of patient characteristics.

Characteristics		Total *N* = 286	Training set *N* = 216 (75.52%)	Testing set *N* = 70 (24.48%)
Age	<15 15–25 >25	71 186 29	66 129 21	5 57 8
		2.5 : 6.5 : 1	3.1 : 6:0.9	0.7 : 8.1 : 1.2
Sex	Female Male	134 152	90 126	44 26
		4.7 : 5.3	2.1 : 2.9	6.3 : 3.7
SES	Low SES High SES	117 169	99 117	18 52
		4.1 : 5.9	2.3 : 2.7	1.3 : 3.7

**Table 2:** Confusion matrix for a validation process of the classification model before dataset preprocessing.

Confusion matrix		Predicted	
		Positive	Negative
Actual	Positive	45	10
	Negative	7	8

**Table 3:** Confusion matrix for a validation process of the classification model after dataset preprocessing.

Confusion matrix		Predicted	
		Positive	Negative
Actual	Positive	53	2
	Negative	4	11

**Table 4:** Quantitative analysis of different segmentation models in MRI images of osteosarcoma.

Model	PRE	REC	IOU	DSC	F1	Parameters	FLOPS
U-Net	0.922 ± 0.09	0.924 ± 0.08	0.867 ± 0.04	0.892 ± 0.04	0.923 ± 0.05	17.26M	160.16G
PSPNet	0.856 ± 0.09	0.888 ± 0.05	0.772 ± 0.04	0.870 ± 0.06	0.872 ± 0.03	49.07M	101.55G
MSFCN	0.881 ± 0.06	0.936 ± 0.03	0.841 ± 0.02	0.874 ± 0.03	0.906 ± 0.05	20.38M	1524.34G
MSRN	0.893 ± 0.03	0.945 ± 0.05	0.853 ± 0.05	0.887 ± 0.03	0.918 ± 0.04	14.27M	1461.23G
FCN-16s	0.922 ± 0.09	0.882 ± 0.06	0.824 ± 0.04	0.859 ± 0.07	0.900 ± 0.08	134.3M	190.35G
FCN-8s	0.941 ± 0.07	0.873 ± 0.05	0.830 ± 0.05	0.876 ± 0.04	0.901 ± 0.04	134.3M	190.08G
FPN	0.914 ± 0.11	0.924 ± 0.07	0.852 ± 0.05	0.888 ± 0.08	0.919 ± 0.07	88.63M	141.45G
UATransNet Residual	0.962 ± 0.03	0.945 ± 0.04	0.922 ± 0.03	0.921 ± 0.04	0.955 ± 0.05	17.9M	161.01G
UATransNet Dense	0.960 ± 0.05	0.941 ± 0.05	0.918 ± 0.02	0.916 ± 0.07	0.950 ± 0.06	18.3M	163.20G

## Data Availability

The data used to support the findings of this study are currently under embargo, while the research findings are commercialized. Requests for data, 12 months after publication of this article, will be considered by the corresponding author.
